# Effect of Narrative Nursing Intervention Based on Targeted Nursing Intervention on Anxiety and Nursing Satisfaction of Patients with Malignant Tumors Undergoing Chemotherapy

**DOI:** 10.1155/2021/4438446

**Published:** 2021-11-30

**Authors:** Huixia Xu, Guoping Xu, Ying Liu, Xuejing Mu, Yang Liu, Haiping Hu

**Affiliations:** ^1^Department of Internal Medicine-Oncology, The Fourth Hospital of Hebei Medical University, Hebei Cancer Hospital, Shijiazhuang, 050011, China; ^2^Department of Urology and Anorectology, Wuhan Xinzhou District People's Hospital, Wuhan 430400, Hubei Province, China

## Abstract

**Objective:**

To explore the effect of narrative nursing intervention based on targeted nursing intervention on anxiety and nursing satisfaction of patients with malignant tumors undergoing chemotherapy.

**Methods:**

120 malignant tumor patients treated with chemotherapy in our hospital from January 2019 to January 2020 were selected as the research objects and randomly divided into group A and group B, with 60 cases in each group. The targeted nursing intervention was performed to group B, and the targeted nursing intervention centering on narrative nursing was performed to group A, so as to compare their distress thermometer (DT) scale scores, depression and anxiety scale scores, Medical Coping Modes Questionnaire (MCMQ) scores, Functional Assessment of Cancer Therapy-General (FACT-G) scores for quality of life, and nursing satisfaction.

**Results:**

After nursing intervention, group A obtained 5.00 ± 1.20 points in the DT score, which were significantly lower than group B (*P* < 0.05); and group A achieved significantly lower depression and anxiety scale scores (*P* < 0.001), better MCMQ scores (*P* < 0.05), and higher FACT-G scores (*P* < 0.05) and nursing satisfaction (*P* < 0.05) than group B.

**Conclusion:**

The targeted nursing intervention based primarily on narrative nursing can greatly reduce negative emotions, alleviate anxiety, and improve confidence in treatment and quality of life for malignant tumor patients undergoing chemotherapy, with higher nursing satisfaction, which should be promoted and applied in the practice.

## 1. Introduction

The pathogenic factors of tumors are complicated. With the changing environment nowadays, the number of patients suffering from malignant tumors worldwide is increasing year by year, and most of them have an insidious onset and are often at the end stage of the disease when diagnosed, at which time chemotherapy has become the first choice to prolong the survival time of patients [1–3]. Chemotherapy, although it suppresses the condition, leads to corresponding adverse reactions and toxic side effects in patients. During the long-term course of chemotherapy, patients tend to have serious psychological burden and negative emotions such as hopelessness, depression, and anxiety that seriously affect their physical and mental health because of body function decline, increasing economic pressure, self-cognitive disorder, and reduced self-efficacy [4–7]. In current practice, the routine chemotherapy nursing mode usually oriented to the completion of a chemotherapy task is often adopted, but its application effect needs to be improved because it is not individually different and the nursing personnel cannot evaluate and intervene on the psychological status of patients. With the increasing attention paid to humanistic nursing, narrative nursing has been gradually applied to the clinic, which mainly refers to the nursing mode that the nursing personnel physically carry themselves into the patient's place by communicating and listening, deeply grasp the actual problems faced by the patient, propose targeted responses to resolve the patient's dilemma, and then alleviate their negative emotions [8–11]. Applying narrative nursing based on targeted nursing is more individually different, which can fundamentally solve the problems raised by the patients with different conditions and of different educational levels, comprehensively improve the psychological nursing effect, and enhance the application value. However, it is still in the immature stage at present. Based on this, to explore the effect of narrative nursing based on targeted nursing intervention on the anxiety and nursing satisfaction of malignant tumor patients undergoing chemotherapy, 120 such patients treated in our hospital from January 2019 to January 2020 were selected for the study, with the results summarized as follows.

## 2. Materials and Methods

### 2.1. General Information

120 malignant tumor patients undergoing chemotherapy treated in our hospital from January 2019 to January 2020 were selected for the study and randomly divided into group A and group B, with 60 cases in each group and no statistical difference in their general information (*P* > 0.05); see Table 1. The study was approved by the Hospital Ethics Committee.

### 2.2. Inclusion Criteria

The inclusion criteria of the study were as follows. (1) The patients or their family members fully understood the study process and signed informed consent; (2) the patients were diagnosed as malignant tumor after examination and had the need for chemotherapy [12]; (3) the DT scores of the patients were more than 4 points [13]; and (4) the estimated survival time of the patients was more than 6 months.

### 2.3. Exclusion Criteria

The exclusion criteria of the study were as follows. (1) The patients had mental problems or were unable to communicate with others; (2) the patients had other organic diseases; (3) the functional status scores of the patients were less than 3 points [14]; and (4) the patients were unclear about their condition [15].

### 2.4. Methods

Targeted nursing intervention was performed to group B with the following specific steps. (1) The nursing personnel should master the detailed personal information of patients, so as to give careful targeted nursing and intervention on routine medication to patients. (2) Malignant tumor patients undergoing chemotherapy usually had a low tolerance, and after multiple times of chemotherapy, they were prone to have unhealthy psychological state because of the decreased body condition and economic status. At this time, the nursing personnel should increase the frequency of communication with patients during chemotherapy, tell patients about the need of chemotherapy, and inform patients about common adverse reactions, thus alleviating the patients' confusion and enhancing their beliefs about treatment; for the patients with more serious negative emotions or a tendency to experience major anxiety or depression, special psychotherapy should be conducted immediately. (3) The targeted diet during chemotherapy for patients was proposed according to their dietary preferences, e.g., more fresh fruits and no durian for breast cancer patients; patients should eat more food such as eggs and fish everyday while reducing the intake of spicy food to avoid CNS irritation. (4) The nursing personnel should carry out environment-targeted care to reduce the effect of noise, smell, temperature, and other factors on patients and encourage patients to maintain a regular pattern of rest to reduce their mental stress.

Targeted nursing intervention centering on narrative nursing was performed to group A, with the following specific steps. (1) Before treatment, the nursing personnel should comprehensively memorize the patients' information and have a one-on-one communication in the form of personal intervention with the patients in a private place, so as to lay a good foundation for targeted nursing. (2) In each chemotherapy cycle, the nursing personnel should communicate with the patients in private three times, of which the content should be proposed according to the actual situation of the patients and in combination with the personal care details, and each communication should not be less than 1 hour and should follow the will of the patients. Instead of enforcing interference with patients who have a low desire for private communication, communication should be transferred to routine nursing in a subconscious manner, thereby elevating the frequency of daily communication with patients. (3) At the first communication, the nursing personnel must combine the psychological characteristics of the patients to establish a good trusting relationship with them, analyze the patients' anxiety and carry out corresponding communication by interpreting the personal data, guide the patients to pour out his or her true thoughts, and encourage the patients to speak up the inner pain and uneasiness. And for the shy patients, the nursing personnel should proactively ask about their living situation in daily chat; the nursing personnel should not be critical to the responses of patients and should only be empathetic by putting themselves in the benefit of patients so that patients would feel that they could rely on the nursing personnel. (4) The nursing personnel should explore and express the problem with the patients and analyze the impact that the problem has on the patients' mind and life; during communication, the nursing personnel should make clear what factors will enhance and weaken the psychological anxiety and the key points that affect the problem, thereby drawing up the targeted nursing programs that suit the remedy to the case. (5) In the communication process, the nursing personnel should discover the good side of the patients' lives and bring the best in life to therapy so that the patients could take control of their own lives again, build up confidence in the treatment, and hold hope for the future. (6) The nursing personnel should extract the information obtained in the communication and apply it in targeted nursing to provide patients with individually different nursing regimens.

### 2.5. Observation Criteria

When issuing questionnaires, the study group gave only simple instructions about the questionnaires and made no other hints. The questionnaires were taken back after filling out by the patients, and the integrity was verified.

1. DT: based on the screening tool for assessing psychological distress, the distress thermometer (DT) was selected to measure distress in patients on a scale of 0–10, with higher levels indicating more distress [16]. The reliability of the screening tool has been confirmed by the domestic and foreign literature.
2. Depression and anxiety scale scores: the Self-Rating Anxiety Scale (SAS) and Self-Rating Depression Scale (SDS) were selected as the scoring basis, with 20 items each and the total maximum score of 100 points. Higher scores indicated that the negative emotion of patients was more serious [17]. The reliability of the scales has been confirmed by the domestic and foreign literature.
3. Medical Coping Modes Questionnaire (MCMQ): it included three coping modes, namely, confrontation, avoidance, and acceptance-resignation, which consisted of different items. The questions for the confrontation worded toward increasing levels, and the questions for the other two dimensions worded toward decreasing levels. The Chinese version of the MCMQ included 20 items and should be filled in by the patients themselves [18]. The reliability of the MCMQ has been confirmed by the domestic and foreign literature.
4. Functional Assessment of Cancer Therapy-General (FACT-G): it stood for the quality of life in cancer patients for the past 7 days, including physical, social/familial, emotional, and functional well-being. On a scale of 0–180 points, the higher scores indicated better quality of life in patients [19]. The reliability of FACT-G has been confirmed by the domestic and foreign literature.
5. Nursing satisfaction: the nursing satisfaction of patients was investigated by the self-proposed scale of our hospital, and the items included the nursing error rate, attitude toward patients, and nursing service quality. On a scale of 0–5 stars, 5 stars indicated fully satisfied, 3-4 stars indicated satisfied, and 2 stars and less indicated dissatisfied. The number of satisfied patients was counted.

### 2.6. Statistical Processing

In this study, data processing software was SPSS 20.0, picture drawing software was GraphPad Prism 7 (GraphPad Software, San Diego, USA), items included were enumeration data and measurement data, methods used were *X*^2^ test and *t*-test, and differences were considered statistically significant at *P* < 0.05.

## 3. Results

### 3.1. Comparison of DT, SAS, and SDS Scores

After nursing intervention, the DT, SAS, and SDS scores of group A were significantly lower than those of group B (*P* < 0.05); see Figure 1.

Figure 1(a) indicates that the DT scores of both groups before intervention were not statistically different (6.30 ± 1.56 vs. 6.32 ± 1.54, *P* > 0.05); and after intervention, group A obtained significantly lower DT scores than group B (5.00 ± 1.20 vs. 5.89 ± 1.52, *P* < 0.05).

Figure 1(b) indicates that the SDS scores of both groups before intervention were not statistically different (59.65 ± 6.65 vs. 59.54 ± 6.52, *P* > 0.05); and after intervention, group A obtained significantly lower SDS scores than group B (45.11 ± 65.32 vs. 51.21 ± 66.35, *P* < 0.05).

Figure 1(c) indicates that the SAS scores of both groups before intervention were not statistically different (55.98 ± 5.98 vs. 55.48 ± 5.68, *P* > 0.05); and after intervention, group A obtained significantly lower SAS scores than group B (40.12 ± 5.69 vs. 50.12 ± 5.65, *P* < 0.05).

### 3.2. Comparison of MCMQ Scores

After nursing intervention, the MCMQ scores of group A were significantly better than those of group B (*P* < 0.05); see Table 2.

### 3.3. Comparison of FACT-G Scores

After nursing intervention, the FACT-G scores of group A were significantly higher than those of group B (*P* < 0.05); see Table 3.

### 3.4. Comparison of Nursing Satisfaction

The nursing satisfaction of group A was significantly higher than that of group B (*P* < 0.05); see Figure 2.

The number of fully satisfied patients in group A and group B was 28 and 18, respectively. The number of satisfied patients in group A and group B was 30 and 32, respectively. The number of dissatisfied patients in group A and group B was 2 and 10, respectively (*X*^2^ = 5.926, *P*=0.015).

## 4. Discussion

Humanity care is the core spirit of the nursing discipline, and empathy is necessary for nursing personnel to perform nursing interventions. Narrative nursing refers to the way in which nursing personnel view the problem through the patients' perspective and discover the key points of individual care to propose targeted care options for the patients that realistically address their distress and problems [20, 21]. Patients with malignant tumors usually need to receive long-term chemotherapy and are overwhelmed by the body suffering caused by the disease, the toxic side effects from chemotherapy, and the time and money spent on treatment. The vast majority of patients undergoing chemotherapy show different degrees of anxiety and depression during treatment, and some even develop into somatic symptoms that adversely affect their prognosis. Scholars Nancy et al. reported that narrative nursing can effectively improve patients' negative emotion and reduce the impact of negative emotions on patients' body condition [22]. Therefore, alleviating their negative emotions is an important part of humanity nursing. In this study, the DT, SDS, and SAS scores of group A were obviously lower than those of group B (*P* < 0.05), indicating that the targeted nursing intervention centering on narrative nursing could create a safe and relaxed face-to-face and one-on-one communication environment for patients so that patients could tell the nursing personnel about their doubts and insecurities and the nursing personnel could help the patients in analyzing their problems, and as a result, the patients were able to view their difficulties through a new angle, gained clearer recognition of the disease, and reduced their anxiety.

In addition, after the targeted nursing intervention focused on narrative nursing, the patients could review their lives, feel their shinning spots in life again, and bring positiveness into the treatment, thereby building up confidence and a stronger attitude toward treatment [23]. Scholars Bradley et al. found that targeted nursing can reduce patients' hostility and enable the patients to experience targeted psychological nursing, promote their trust in nursing personnel, and increase their positivity over treatment [24]. The study results showed that, after intervention, group A achieved 22.65 ± 2.68 points in the MCMQ score, which were significantly better than group B (*P* < 0.05), proving that such nursing mode could change the anxious state of malignant tumor patients undergoing chemotherapy for them to take control of their own lives again and fully activate their positive quality; hence, patients in group A faced their difficulties with a more positive attitude.

Compared with group B after nursing intervention, group A obtained a significantly higher score in FACT-G (*P* < 0.05), a scale to evaluate the quality of life of cancer patients, which was consistent with the findings of Beesley and others. In their study, patients in the experimental group received the targeted nursing intervention centering on narrative nursing, and patients in the control group were given the targeted nursing intervention, and it was concluded that the total FACT-G scores of the experimental group were 74.12 ± 12.56 points, which were remarkably higher than those of the control group (*P* < 0.001) [25], verifying the fact that the targeted nursing intervention focused on narrative nursing had a positive effect on improving the quality of life in patients and comprehensively promoting the daily life status. With better psychological status and quality of life, the anxiety would be alleviated; hence, the nursing satisfaction of group A was significantly higher than that of group B (*P* < 0.05), indicating that such nursing mode could effectively lower the possibility of nurse-patient dispute and improve the nursing quality.

In conclusion, the targeted nursing intervention based primarily on narrative nursing can greatly reduce negative emotions, alleviate anxiety, and improve confidence in treatment and quality of life for malignant tumor patients undergoing chemotherapy, with higher nursing satisfaction, which should be promoted and applied in the practice.

## Figures and Tables

**Figure 1:** Comparison of DT, SAS, and SDS scores ($\bar{X}$ ± *s*, points). (a) DT scores. (b) SDS scores. (c) SAS scores. The horizontal axes from left to right indicated before and after intervention, and the vertical axes indicated the scores (points); the black areas indicated group A, and the gray areas indicated group B.

**Figure 2:** Comparison of nursing satisfaction. Note: in Figure 2, the black area indicated fully satisfied, the dark gray area indicated satisfied, and the light gray area indicated dissatisfied; the left image indicated group A, and the right image indicated group B.

**Table 1:** Comparison of general information.

Group	Group A (*n* = 60)	Group B (*n* = 60)	*X* ^2^/*t*	*P*
*Gender*			0.034	0.853
Male	25	26		
Female	35	34		
*Age (years)*				
Range	32–74	33–74		
Mean age	41.21 ± 6.20	41.23 ± 6.21	0.018	0.986

*Tumor category*				
Lung cancer	10	11	0.058	0.810
Breast cancer	12	11	0.054	0.817
Digestive tract malignant tumor	12	13	0.051	0.822
Others	26	25	0.034	0.853

*Disease stage*				
I	12	11	0.054	0.817
II	30	30	0.000	1.000
III	18	19	0.039	0.843

*Basic diseases*				
Diabetes	12	11	0.054	0.817
Hypertension	15	14	0.046	0.831
Coronary heart disease	8	9	0.069	0.793
Lung disease	8	10	0.261	0.609

*Educational level*				
Junior high school or lower	12	10	0.223	0.637
Senior high school	28	30	0.134	0.715
College or higher	20	20	0.000	1.000

*Monthly income (yuan)*				
>3000	24	23	0.058	0.810
≤3000	36	37	0.035	0.852

**Table 2:** Comparison of MCMQ scores after intervention ($\bar{X}$ ± *s*, points).

Group	*n*	Confrontation	Avoidance	Acceptance-resignation
Group A	60	22.65 ± 2.68	14.98 ± 2.65	9.21 ± 2.15
Group B	60	18.98 ± 2.68	15.98 ± 2.35	12.65 ± 2.54
*t*		7.501	2.187	8.007
*P*		0.000	0.031	0.000

**Table 3:** Comparison of FACT-G scores after intervention ($\bar{X}$ ± *s*, points).

Group	Total scores	Physical well-being	Social/familial well-being	Emotional well-being	Functional well-being
Group A	72.65 ± 12.11	20.11 ± 2.65	16.98 ± 2.65	17.14 ± 3.65	18.10 ± 2.65
Group B	64.32 ± 12.54	17.10 ± 5.65	14.21 ± 4.20	14.20 ± 2.68	15.98 ± 3.15
*t*	3.701	3.736	4.321	5.029	3.989
*P*	0.000	0.000	0.000	0.000	0.000

## Data Availability

The data used to support the findings of this study are available from the corresponding author upon reasonable request.
